# Engineering Education Understanding Expert Decision System Research and Application

**DOI:** 10.1155/2022/9662301

**Published:** 2022-05-02

**Authors:** Huajie Ye, Cuifeng Li

**Affiliations:** Zhejiang Business Technology Institute, Ningbo 315012, Zhejiang, China

## Abstract

Engineering education is based on technical science and aims at training engineers who can transform science and technology into productive forces. In recent years, due to the emergence of new technology revolution, engineering science and production technology have achieved new development, and higher engineering education is also facing new challenges. Engineering education is to cultivate talents in an international environment and update the traditional engineer training model from the aspects of educational philosophy, mode, goal, approach, and means. The author believes that in the process of exploring the new talent training model, we must first change the educational concept and correctly understand and deal with various relationships in engineering education. To solve various decision-making problems in engineering construction, this study introduces the concept of engineering education certification under the background of new infrastructure and engineering education certification, analyzes the current situation and existing problems of engineering education understanding in recent years, and carries out reform and exploration from different aspects. The achievements in engineering education are analyzed. The engineering education project is analyzed and researched using the engineering decision-making scheme. It can be seen from the experimental analysis that the method has a good effect.

## 1. Introduction

With the advancement of science and technology and the change in the international environment, the training mode of engineering education talents in engineering colleges in my country has become more and more unsuitable for the current situation. To reform the traditional engineering education talent training model, the most urgent task is to change the educational concept and correctly understand and handle the relationship between one-time education and lifelong education, professional education and quality education, school education and factory-enterprise cooperative education, and theoretical education and practical education [1–3]. China's higher engineering education mainly learns and learns from the model of the former Soviet Union, strengthens professional counterpart education, and trains professional talents for industrial construction. A professional curriculum system should be affirmed. At a time when China's productivity, technology, and culture are very backward, and all walks of life are waiting for development, all kinds of professional talents are urgently needed, and the country should develop scale according to a strict planning system [4–6]. The role played is considerable. The various professionals we have cultivated have made outstanding contributions to the economic development of the motherland on various fronts, and in this teaching system, we inherit and retain scientific rigor. The systematic tradition has played a very important role in improving the quality of education on a large scale. However, with the passage of time, it is difficult for the overly detailed majors to meet the needs of modern scientific and technological development and social and economic development, and the defects of professional education are constantly exposed. The specific manifestations are that the division of disciplines and majors is too detailed, the knowledge of students is too specialized and too narrow, and it cannot adapt to the characteristics of interdisciplinary, infiltration, and high integration of modern engineering practice and it is difficult to undertake the organization and management tasks of modern engineering [7–10].

In recent years, the problems of engineering education have become more and more complex and continue to transcend pure scientific and technological problems. Engineering and social politics, economy, structure, ecology, morality, etc., are increasingly connected. The students trained are no longer “rough” engineers in the traditional sense, but should be high-quality modern engineers with modern engineering awareness, understanding of engineering background and environment, mastering the latest engineering knowledge and technology, and adapting to modern engineering needs [10–14]. In the stage of engineering education, in addition to learning certain professional theoretical knowledge, carrying out certain preparatory training for social practice, and laying a solid foundation for them to go to the society, go to work, and play a certain role in social activities, they also need to strengthen students. The formation of students' world outlook, outlook on life, values, and moral values needs positive and correct guidance; their independence, enthusiasm, autonomy, and creativity need to be further strengthened; and their political ideology, morality, and spiritual qualities need to be further strengthened. Sublimation, its humanities, and social knowledge need to be further expanded; the communication, communication and unity, and cooperation skills required for social life need to be cultivated and exercised; and its literary and artistic accomplishment, temperament, and oral and written expression skills need to be further improved [15–18]. That is to say, from the perspective of big science and big engineering, it is necessary to carry out extensive learning and comprehensive quality training on society, culture, economy, law, environment, management, communication, and other knowledge that are essential for future engineers.

In fact, the training and improvement of the engineering practice ability of engineers are ultimately completed in the enterprise. Some modern enterprises in China, such as Baosteel Group, take three-year indefinite positions for college students who have newly entered the factory—“One year to strengthen, two years to enrich, three years.” The method of “diversion” is used to carry out training, strengthen the professional knowledge of college students, and make them more adaptable to the needs of enterprises. However, there are still a large number of small- and medium-sized enterprises and township enterprises in our country. They require college students to play a role in the factory immediately. I hope that graduates have strong engineering practice ability. Facing the imbalance of regional development and the level of enterprise development, the students we train must have strong adaptability. This is the national condition of China's higher engineering education. Although this problem is in the world, it will be encountered in all countries, but it is particularly prominent in China [19–22]. Due to the lack of a mechanism for undertaking engineering training in China's industrial system, most factories do not have specialized training institutions and trainers. Modern production also makes it difficult for students to directly contact engineering objects. To cultivate students' engineering practice ability, engineering colleges have established school-run enterprises in the school, but many of these school-run enterprises are of unknown nature and low level of management and management, and it is difficult to compare with social enterprises. With the deepening of the reform of the internal management system in colleges and universities, school-run enterprises are separated from schools and become relatively independent and self-operated enterprise units, but their engineering environment is completely different from the real engineering environment of large- and medium-sized enterprises. Each major has a corresponding school-run enterprise as an on-campus practice base. Therefore, school-enterprise cooperative education should become an important supplementary form of current higher engineering education [23–26].

School-enterprise cooperative education requires the joint efforts of schools and enterprises. However, due to the lack of corresponding rules and regulations in this area in my country, many colleges and production systems have not achieved positive results in “colleges are oriented to enterprises, and enterprises rely on education and technology.” Therefore, on the one hand, the government and relevant state departments should actively support and assist school-enterprise cooperative education, and through some administrative and legislative means, a group of large- and medium-sized enterprises is selected with better benefits, a certain amount of funds is invested, or certain preferential policies are implemented. A batch of production practice and engineering practice bases is built, and the peripheral environment required for engineering education is effectively improved; various forms of contact and cooperation with enterprises are carried out, from point to face, and a new path with its own characteristics is persevered and found to comprehensively improve the quality of engineering education.

With the wide application of computers and intelligent equipment in my country, my country has begun to conduct research on the cognition of expert decision-making systems in engineering education. A large number of studies have been carried out, and rich results and experience have been obtained, which has made outstanding contributions to the development of engineering education cognition in my country. In recent years, although the promotion of relevant expert systems has been carried out successively, it is still difficult to query and retrieve professional data. In addition, the workload of summarizing various test results is very large, which will consume a lot of resources. Looking back at the process of implementing expert system cognitive technology in my country, although the results have been remarkable, there are some problems that cannot be ignored, the most important of which is that this technology has not been deeply and widely used. According to the research and investigation, so far, there are very few cases that can actually achieve accurate decision-making. In most cases in my country, the decision-making system is still used for reference, the acceptance of new technologies is still not significantly changed, and traditional phenomena are still common. Although there are many reasons for this situation, it is inevitable to promote engineering education cognition through computer expert system. This study designs and verifies the remarkable effect of expert decision-making system in engineering education cognition.

This study is divided into 5 sections. Section 1 describes the purpose and direction of the research. Section 2 is the analysis of systematic research methods. Section 3 is system requirement analysis and overall design. Section 4 is the concrete realization of expert decision-making system. Section 5 is summary and outlook.

The research contributions of the study are as follows:

1. This study introduces the concept of engineering education certification in the context of new infrastructure and engineering education certification.
2. The current situation and existing problems of engineering education cognition in recent years are analyzed, and various aspects for reform and exploration are proposed.
3. The achievements of engineering education are analyzed. The engineering education project is analyzed and researched using the engineering decision-making scheme.

## 2. Analysis of Current Situation of Cognition in Engineering Education

Under the background of engineering education certification, the status quality of engineering cognition practice can no longer fully meet the ability requirements of engineering certification. Like most of the current undergraduate schools, the school's understanding of internships is a group visit to the internship site. Through the students' perceptual understanding, they have a preliminary understanding of the composition of the building, the building function, the building structure and building materials, and the layout of the construction site. It is difficult to be satisfied with the practice process and results, which violates the “student-oriented” evaluation concept of engineering education certification, and it is difficult to meet the basic requirements of engineering certification for competence.

### 2.1. Difficulty in Contacting the Internship Site

Traditional engineering recognizes that the practice site is the construction site, and various reasons make it more and more difficult to contact the practice site. Due to the engineering awareness practice, there are many special requirements for the practice site, such as not too far from the school, having completed or just completed a certain process, practice safety, etc. The regulatory authorities have stricter requirements on construction safety, and construction companies are reluctant to accept students for internships out of safety concerns. In recent years, air pollution control has caused many areas to require construction sites to shut down for some months. For the convenience of description, the reasons can be described as follows:

(1) $$\begin{array}{c} I\left(m\right)=\left\{\begin{array}{cc} 0, & \text{pollution}<\text{threshold,}\\ 1, & \text{pollution}\geq \text{threshold,} \end{array}\right. \end{array}$$

where pollution(*m*) is the *m*th month pollution of the current year. Threshold is the default setting to determine whether the pollution is accepted in the specific month. If *I*(*m*)=1, we reject to internship; otherwise, we can accept students for internship.

### 2.2. Great Safety Hazard

First of all, due to the particularity of the construction site work, there are many open air operations and high-altitude operations, poor construction environment and working conditions, many types of work involved, and many cross-operations, and safety production accidents occur from time to time. Secondly, when students arrive at the construction site for the first time, they lack awareness of the potential safety hazards on the construction site, and they do not pay attention to their own and others' safety, which can easily lead to safety accidents. Finally, as the internship site is getting farther and farther from the school, the safety of students on the way to the internship has also become a factor that must be considered as follows:

(2) $$\begin{array}{c} D_{t+1}=D_{t}+R_{t+1}. \end{array}$$

All the above variables are nonnegative variables, where *D*_*t*+1_ is the index of danger of *t*+1 period; *R*_*t*+1_ is the potential danger factor in the period *t*+1, the equation means that the danger of current equals to the danger of former time and the potential danger factor of current time.

### 2.3. Internship Mode Is Single

The traditional practice is just to visit the construction site blindly, and the mode is single. With the rapid development of new technologies such as prefabricated, BIM, VR, and the country's layout of “new infrastructure,” the construction industry has begun a technological revolution characterized by informalization, assembly, and intelligence. If the content and mode of understanding internships do not keep pace with the times, the content of internships will be out of touch with the development of the construction industry, and students will not be able to meet the requirements of the professional certification standards to understand the current status and trends of the frontier development of the major.

### 2.4. The Teaching Effect Is Poor and the Students Gain Little

In traditional cognition practice, professional teachers organize and lead students to visit the construction site. While visiting, they are explained by engineers or leading teachers. The whole internship process of students is very passive, and they can only “listen and watch” and have no active consciousness. At the same time, because the construction site environment is not suitable for teaching, many students cannot listen carefully. When students first arrive at the internship site, they often have a strong sense of freshness. During the internship, they will feel that the difficulty is relatively low. The internship reports of some students reflect that the internship results and gains are small, and the content is fragmented, and unspecific. It looks like a running account and lacks breadth and depth. This teaching mode emphasizes the teacher as the center, which is completely cramming teaching, and the students' practical ability cannot be exercised and improved at all.

### 2.5. The Assessment Method Is Not Scientific

Although the final grades of the internship will refer to the discipline and speech performance of the students during the internship, the assessment method is generally a “one-time assessment,” and the score is only based on the internship report, which cannot mobilize the students' enthusiasm for the internship at all. At the same time, because the content of students' practice is basically the same, students are opportunistic, and the phenomenon of the same practice report is very serious. Teachers cannot grasp the actual situation when grading, nor can they reflect the distinction of assessment.

## 3. Systematic Research Method Analysis

### 3.1. Method Used by the System

#### 3.1.1. Effect Function Method

To use this method, we must first establish an experiment on engineering education cognition and study its data. Through the obtained effect equation, we can estimate the specific cognition and decision-making inference and provide a reference for accurate decision-making. Since this method is a mathematical method based on experiments, there is no need to resort to physical or chemical means to estimate the actual decision effect. The relationship between the decision result and the influencing factors is called the decision effect, and the mathematical formula reflecting the relationship is called the effect function or the effect equation. The effect function is generally represented by a quadratic polynomial as follows:

(3) $$\begin{array}{c} y=a+bx+cx^{2}. \end{array}$$

This is the single-element effect function expression. In the formula, *x* represents the decision-making speed and *y* represents the decision-making effect after applying a specific decision; *a*,  *b*,  *c*  are the regression coefficients, where *a* represents the effect of not applying the corresponding decision; *b* represents the magnitude of the positive decision-making effect; and *c* is the curvature, representing that after the decision was applied, the effect showed a downward trend. The functional expression of the two-element effect is as follows:

(4) $$\begin{array}{c} y=a+bx+cx^{2}+dz+ez^{2}+fxz, \end{array}$$

where *y* represents the decision effect under two influencing factors; *x*,  *z* represent these two different decision factors; and  *a*,  *b*,  *c*,  *d*,  *e*,  *f*  are partial regression coefficients, where *a* is the actual effect when no decision factor is applied, *b*, *d* represent the growth effect of the two factors, respectively, *c*, *e* represent the descending curvature when the decision factor is applied, and *f* is the interaction effect of the two factors, which can be obtained by statistical methods.

#### 3.1.2. Factor Balance Method

The component balance method is also called the total cognitive target method. The relevant parameters involved include target total, influencing factors, and relationship influencing factors. The total amount of targets is the total amount of expert decision-making on educational cognition. The determination of the decision by the expert decision system can be accomplished by different calculation methods.

The component balance method calculates the factor variables by calculating the difference between the specific implementation amount and the actual feeding amount of different factors to achieve the decision goal. The calculation formula is as follows:

(5) $$\begin{array}{c} Q\_diff=\frac{Tar-\text{Povide}}{\text{Content}*\text{Vilidation}},\\ Q_{imp}=\frac{\left(Tar-\text{baseline}\right)*{\text{absolve}}_{\text{unit}}}{\text{Content}*\text{Vilidation}}. \end{array}$$

The effective correction coefficients for different factors are based on the effectiveness of the effective factors to calculate the influence. The unit of measurement of general factors is %, and the conversion factor of 0.15 can be obtained by converting the influence of each unit into %. The calculation formula of this method is as follows:

(6) $$\begin{array}{c} Q_{imp}=\frac{{\text{absolve}}_{\text{unit}}*{\text{Target}}_{\text{pro}}-\text{content}*0.15*\text{revise}\_\text{parameters}}{\text{Content}*\text{Vilidation}}. \end{array}$$

The calculation of the nutrient requirements for the target yield uses the whole-plant nutrient analysis method, that is, the product of the nutrient value required by the actual yield per 100 kg of mature crops and the target yield.

(7) $$\begin{array}{c} \text{Target\_content}=\frac{\text{Target\_pro}}{100}*\frac{\text{Content}}{100\text{\%}}\text{.} \end{array}$$

The calculation of the utilization rate of fertilizer in the current season must first determine the nutrient supply amount of the fertilizer, that is, the difference between the actual nutrient absorption of a crop in the fertilized area and the actual nutrient absorption of the crop in the non-fertilized area, and this value is divided by the applied nutrient. The percentage of nutrient content of the fertilizer can be used to obtain the seasonal utilization rate of the fertilizer as follows:

(8) $$\begin{array}{c} \text{Utilization}\left(\%\right)=\frac{{\text{Absolve}-\text{absolve}}_{\text{lackzone}}}{{\text{Gross}}_{imp}*\text{Content}}*100\text{\%.} \end{array}$$

### 3.2. Comparison of Advantages and Disadvantages of Methods

The effect function method can visually express the single and comprehensive effects of relevant factors on yield, that is, the different yield-increasing effects of single-element fertilizers on specific crops or the synergistic effects of co-application of multiple fertilizers. The higher the degree, the more appropriate to the actual situation. However, the disadvantage of this method is that it has strong limitations and requires a large number of test points to be arranged on plots with different soil types, climates, farming methods, and other conditions. Even in the same area, the previous experimental data and results cannot be reused, and changes in various factors will change the functional relationship, and repeated use will seriously affect the accuracy of fertilizer calculation. This method not only needs to accumulate the experimental data of previous years but also needs to carry out complicated mathematical operations, so it is not suitable for ordinary farmers, and it is very difficult to popularize the technology.

The nutrient abundance index method was once a recommended fertilization method widely used in the world. It is a formula fertilization method advocated in most areas of my country at this stage. The features are as follows: this fertilizer method is a systematic fertilizer determination method, and the specific implementation steps include establishing local soil nutrient abundance indicators, determining the recommended soil fertilizer amount according to the indicators, and detecting the nutrient value of the soil that needs to be fertilized. In the practical application of this method, as long as the soil nutrient value of a certain area is measured, the nutrient grade is obtained by weighted calculation, and finally the recommended application amount of a certain crop and certain fertilizer is determined according to the grade. The difficulty of this method lies in properly grading the nutrient content of the soil and designing fertilization recommendations corresponding to different nutrient levels. Its advantages of strong intuition, simplicity, and convenience are suitable for the current agricultural situation, but its poor accuracy is not conducive to the long-term development of agriculture.

The biggest advantage of the factor balance method is that the concept is clear and the calculation is simple and fast. Because this method can estimate the reasonable amount of fertilizer application by means of soil testing, it is easier for farmers to master. However, because the material system such as soil has great buffering property, its nutrient content will change with the change in crop growth and environmental conditions, so that the entire soil system always maintains a dynamic balance. The measured value of soil nutrients is only a relative value and cannot reflect the actual supply of soil. The correction coefficients are quite different for different regions and different crops, so this method requires a lot of parameters, so it is difficult to control the accuracy of the calculation, but in the case of field trials and accurate parameters, its agricultural practicability is very high.

### 3.3. Technology and Tools for System Development

ADO.NET (Active Data Objects) is Microsoft's solution to data access problems in .NET. It provides ASP.NET and Windows Forms applications with consistent access to data sources such as Microsoft SQL Server and data sources exposed through OLEDB and XML. Applications can connect to data sources through ADO.NET for data acquisition, manipulation, and update operations. ADO.NET includes objects described as follows:

1. The Connection object provides functions such as the connection between the system and the data source.
2. The Command object can operate the data of the data source by executing the SQL, including reading, inserting, deleting, and updating the data.
3. The Data Reader object can read data from the data source to the local, but does not assume the responsibility of saving the data, and requires the user to manually close the connection to the database, so it is not a data structure, but a high-level encapsulation of network communication components.
4. The Data Adapter object is the bridge between the data source and the data set, which can be used to fill the data set or data table, that is, to load the data into the memory.
5. Data Set object, with a disconnected data access mechanism, the data reside in the memory and can also directly perform retrieval, insertion, modification, deletion, and other operations on these data.

Database technology is the core technology of computer information system and the key technology of computer-aided data management. By studying how to acquire, store, organize, and process data, it solves the problem of organization, management, and storage of large amount of data in information management. Therefore, the essence of the database system is to reduce the redundancy of data storage, realize the sharing of data, organize and store the data effectively, and ensure the security of the data. Data processing is realized through theoretical research. In general, a database is an application software for research data management.

SQL Server 2008 can store structured, semi-structured, and even unstructured information directly into the database, and then, management, analysis, and processing operations are performed on it. Usually, data can be stored on any information device, from data servers to desktop computers and even mobile devices, and the data in the database can be managed anytime and anywhere. In addition, SQL Server can use databases in custom applications developed using Microsoft.NET and Visual Studio Development tools, including data in service-oriented architecture (SOA) and business processes through Microsoft BizTalk Server. Any user can obtain the corresponding data from the database through the information management tool.

This section mainly briefly introduces the technologies and tools involved in the system. Firstly, various methods and calculation formulas are introduced, and their advantages and disadvantages are analyzed. Secondly, it introduces the software development technology and tools of the system, as well as the core modules and related protocols used in the hardware part.

## 4. System Requirements Analysis and Overall Design

### 4.1. Demand Analysis

The quality of the decision-making system depends not only on whether the technology used is advanced, whether the system structure is reasonable, and whether the functions are perfect but also on whether the system can meet the requirements of users. This requires developers to be familiar with the actual situation before system development. Must understand the requirements and analyze the feasibility of all aspects of the system in detail. My country's engineering education cognition department has insufficient hardware facilities and a limited professional level of technical and scientific personnel, so the system must be guaranteed in terms of professionalism and operability.

Most of the current software systems focus on information management. Through the analysis of the principle and effect of Kriging interpolation, the selection of the best fitting model of Kriging interpolation is realized, and the spatial data processing is designed to realize the calculation of soil fertilizer supply. To combine the real-time data processing of soil monitoring instruments, this study designs a computer system based on .NET technology and database technology that is convenient for users to use fertilization decision-making as the main function. The system needs to be able to easily manage data, including data addition, modification, deletion, and query, and also needs to quickly import and export a large amount of data. Permission management for different user services can ensure efficient system work and maintenance. To cooperate with the data collection of soil nutrient detection equipment and realize the rapid transmission of decision-making information, it is also necessary to realize the rapid transmission of data. The decision-making function needs to meet the actual needs of educational cognition, provide reasonable calculation of cognition and recommendation of methods, and, on this basis, add the system's unique appropriate recommendation decision-making, benefit analysis, and deficiency judgment functions.

### 4.2. Overall System Design

#### 4.2.1. System Design Principles

System design principles are used to regulate the design and development process of a system. The main user-oriented system of this system is education and cognitive workers, but it also has a certain role in assisting decision-making for engineering education students. Therefore, in the design process of the system, it should not only be based on the principles of standardization and practicality but also provide users at different levels different application interfaces. At the same time, it is also very important to improve the performance of the system.

#### 4.2.2. System Design

The functions of the expert decision-making system include basic information management, soil information processing, expert information query, database management, and user and system management. These functional modules include multiple subfunctional modules, such as the basic information management module including basic crop information management, fertilizer basic information management, mathematical model management, and experimental data management; the soil information processing module includes comprehensive fertility evaluation and suitable crop decision-making, and soil testing formula assists decision-making and deficiency judgment. The user and system management module implements the addition, modification and deletion of system users, and permission management; the database management module includes database backup and restoration and Excel import and export, as shown in Figure 1.

The overall structure design diagram of the system shown in Figure 1 comprehensively shows the decision-making process of the engineering project. The rationality of system function module design depends on the understanding of requirements analysis and user operation business process. Therefore, it is necessary to have an in-depth understanding and analysis of the system business process before the function module design. The business process of this system is shown in Figure 2.

Figure 2 introduces the business flow chart of the engineering project and introduces and analyzes the engineering project from each link.

#### 4.2.3. System Module Composition and Function Introduction

*(1) System Management Module*. The function of the system management module is to provide users with basic system operations, including user login, user registration, password modification, user authority modification, and re-login functions. This module is available to all registered users, and the corresponding functions can be used as long as a simple registration is performed.

*(2) Basic Information Management Module*. The basic information management module realizes the quick management of the knowledge base information on which the expert decision-making system is based. The update function of this module can only be operated by data administrators and system administrators, and ordinary registered users can only perform simple query and browsing. This module can improve the accuracy and real-time performance of expert decision-making results by updating various parameters. The detection data module mainly deals with the import and query of data, including serial data reception and data reception based on UDP protocol.

*(3) Information Processing Module*. The information processing module realizes the decision processing function of the system, as shown in Figure 3. The essence of the lack of prime judgment module is data query and simple reasoning.

*(4) Expert Information Query Module*. This module is a database retrieval module, which is a quick query and browsing of expert knowledge or decision-making data stored in the system implemented in combination with the database.

*(5) Database Management Module*. The database management module is to facilitate the management of data in the database. Due to the differences in the level of engineering education in different places, the cognitive level will be different. This module can realize the rapid import and export of large amounts of data, providing support for the convenience of system data maintenance, the accuracy of decision-making, and the extensive application. The system also includes some other useful functions, including a calculation module for factor determination, cognitive level assessment and expert utilization, and a screen capture module [25].

### 4.3. The Concrete Realization of Expert Decision-Making System

For the Pearson correlation coefficient between two variables, its mathematical definition is the quotient of the covariance and standard deviation between the two variables; that is,

(9) $$\begin{array}{c} \rho_{XY}=\frac{\text{Cov}\left(X,Y\right)}{\sigma_{X}\sigma_{Y}}=\frac{E\left(\left(X-\mu_{x}\right)\left(Y-\mu_{y}\right)\right)}{\sigma_{X}\sigma_{Y}}. \end{array}$$

The coefficient defined by the above formula (10) is generally called the overall correlation coefficient. The actual result is the sample correlation coefficient. The covariance and standard deviation need to be estimated based on the sample, which is generally expressed as *r*, and its mathematical definition is as follows:

(10) $$\begin{array}{c} r=\frac{\sum_{i=1}^{n}\left(X_{i}-\overset{-}{X}\right)\left(Y_{i}-\overset{-}{Y}\right)}{\sqrt{{\sum_{i=1}^{n}\left(X_{i}-\overset{-}{X}\right)}^{2}}\sqrt{{\sum_{i=1}^{n}\left(Y_{i}-\overset{-}{Y}\right)}^{2}}}, \end{array}$$

where $\overset{-}{X}$ and *σ*_*X*_ are the sample mean and the sample standard deviation, respectively.

It can be seen from the above formula that this formula can only be used for offline algorithms because it needs to be obtained first. If an online algorithm for real-time analysis needs to be designed, a certain derivation of the above two formulas is required. The derivation steps are omitted below, and the equivalent conclusions are given directly:

(11) $$\begin{array}{c} \rho_{XY}=\frac{E\left(XY\right)-E\left(X\right)E\left(Y\right)}{\sqrt{E\left(X^{2}\right)-{\left(E\left(X\right)\right)}^{2}\sqrt{E\left(Y^{2}\right)-{\left(E\left(Y\right)\right)}^{2}}}},\\ r=\frac{n\sum x_{i}y_{i}-\sum x_{i}\sum y_{i}}{\sqrt{n{\sum x_{i}}^{2}-{\left(\sum x_{i}\right)}^{2}}\sqrt{n{\sum y_{i}}^{2}-{\left(\sum y_{i}\right)}^{2}}}. \end{array}$$

The expert decision-making subsystem needs to support decision-making knowledge management and provide multidimensional model evaluation knowledge base function. Taking knowledge as the unit, through machine learning or manual analysis of the input operating characteristic data, new evaluation modes are discovered, multidimensional evaluation knowledge is established, and knowledge management is carried out. In the process of applying the system evaluation and optimization suggestion function to perform the system evaluation, the multidimensional mode evaluation decision strategy output by the multidimensional mode evaluation knowledge base function will be used to support the system evaluation process and optimization proposal process to form the final evaluation report [26].

### 4.4. Expert Decision-Making System Testing

Software testing is a very important step in the software development process, and comprehensive testing can ensure the robustness and perfection of the system. This section will focus on analyzing and designing system tests according to user requirements, designing test cases for the object control layer of this system, conducting functional tests, and analyzing the test results.

Figure 4 shows the cognitive proportion of decisions made by expert decision-making systems from different perspectives and shows the sources of information for these decisions when making cognitive decisions. It can be seen from the figure on the left that the decision-making sources of the expert system mainly include three parts: the technical angle, the economic angle, and the humanistic angle and other different aspects. As can be seen from the figure on the right, the sources of support for decision-making mainly include friends, family members, classmates, and the Internet and social networks. Among the sources, technology accounts for 26%, economics accounts for 30%, and humanities and other sources account for 35% and 9%, respectively. The source of cognitive experience is mainly obtained from experts, accounting for 32%, and 41% of relatives, friends, and classmates are also very important.

Figure 5 shows the composition of decision ratios in the three stages of pre-decision, in-decision, and post-decision for 4 individual units of varying degrees from the world to different regions. As can be seen from the figure, there are many decision support methods before decision-making. The smaller the individual unit, the richer the decision-making. During the decision-making period, expert decision-making means are in the majority, and the specific performance is as follows: analyzing multiple evaluation indicators to make the final decision. An important finding is that when the individual units are large, especially at the global level, the type of decision support is relatively single. It can be seen from Figure 5 that the decision-making results in the decision-making stage of the method in this study are more effective and more operable.

In this section, test cases are designed according to the requirement analysis, and the main functions of the expert decision-making system are verified. It mainly includes many functions in three parts: knowledge learning, knowledge management, and analysis and optimization. Due to the relative lag in the development of other modules in the performance evaluation system, the interaction between the systems is basically in the form of test piles, and the Web part that interacts with users only checks and verifies the predefined interface data, but in general, the expected effect is finally achieved, and the functional requirements of the demand analysis are realized.

## 5. Conclusion

The limitations of the adaptability of existing software analysis tools have led to the failure of many projects to operate normally. The research in this study is based on this analysis and research, taking into account the actual work scenario, to provide a better user experience. Expert decision-making systems still need to work hard to improve their analytical capabilities in several directions: just locating fine-grained problems with insufficient CPU resources and deploying too many processes are still not enough to solve and fix problems quickly. To further enrich the semantics of analysis, it is necessary to go deep into the bottom layer and use probes, logs, and other means to link performance indicators with specific code, network, and database operations to locate application bottlenecks. At the same time, in the current environment, it is very common to deploy multiple applications on a single machine. However, the currently collected information is collected and analyzed for the entire single machine and does not distinguish how many resources each application occupies. The next plan should be to refine resource utilization to process granularity, link each analysis with specific applications, and solve the problem of single-machine multi-application problem location. Finally, current application deployments tend to be clustered. The decision-making system designed in this study supports multi-machine deployment, but the performance analysis part still lacks the logic of multi-machine information collection and cooperative processing, which is the direction of future research.

## Figures and Tables

**Figure 1:** System overall structure design diagram.

**Figure 2:** Business flowchart.

**Figure 3:** Information process module.

**Figure 4:** The recognition of system on different aspects.

**Figure 5:** Role of expert decision-making in different periods of decision-making.

## Data Availability

The data used to support the findings of this study are available from the corresponding author upon request.

## References

[1] March J. G. (1994). *Primer on Decision Making: How Decisions Happen*.

[2] Slovic P., Lichtenstein S., Fischhoff B. (1988). *Decision Making*.

[3] Duan Y., Edwards J. S., Dwivedi Y. K. (2019). Artificial intelligence for decision making in the era of Big Data - evolution, challenges and research agenda. *International Journal of Information Management*.

[4] Herrera-Viedma E., Palomares I., Li C.-C. (2020). Revisiting fuzzy and linguistic decision making: scenarios and challenges for making wiser decisions in a better way. *IEEE Transactions on Systems, Man, and Cybernetics: Systems*.

[5] van Dijk E., De Dreu C. K. W. (2021). Experimental games and social decision making. *Annual Review of Psychology*.

[6] Marchau V. A. W. J., Walker W. E., Bloemen P. J. T. M., Popper S. W. (2019). *Decision Making under Deep Uncertainty: From Theory to Practice*.

[7] Dos Santos P. H., Neves S. M., Sant’Anna D. O., Oliveira C. H. d., Carvalho H. D. (2019). The analytic hierarchy process supporting decision making for sustainable development: an overview of applications. *Journal of Cleaner Production*.

[8] Xiao F., Cao Z., Jolfaei A. (2021). A novel conflict measurement in decision-making and its application in fault diagnosis. *IEEE Transactions on Fuzzy Systems*.

[9] Orlove B., Shwom R., Markowitz E., Cheong S.-M. (2020). Climate decision-making. *Annual Review of Environment and Resources*.

[10] Pieterse A. H., Stiggelbout A. M., Montori V. M. (2019). Shared decision making and the importance of time. *JAMA*.

[11] Yang M., Nachum O. Representation matters: offline pretraining for sequential decision making.

[12] Kay J., King M. (2020). *Radical Uncertainty: Decision-Making beyond the Numbers*.

[13] Leicht-Deobald U., Busch T., Schank C. (2019). The challenges of algorithm-based HR decision-making for personal integrity. *Journal of Business Ethics*.

[14] Lantos J. D. (2018). Ethical problems in decision making in the neonatal ICU. *New England Journal of Medicine*.

[15] Bousdekis A., Lepenioti K., Apostolou D., Mentzas G. (2021). A review of data-driven decision-making methods for industry 4.0 maintenance applications. *Electronics*.

[16] Légaré F., Adekpedjou R., Stacey D. (2018). Interventions for increasing the use of shared decision making by healthcare professionals. *Cochrane Database of Systematic Reviews 2018*.

[17] Jamwal A., Agrawal R., Sharma M., Kumar V. (2021). Review on multi-criteria decision analysis in sustainable manufacturing decision making. *International Journal of Sustainable Engineering*.

[18] Bishop S. J., Gagne C. (2018). Anxiety, depression, and decision making: a computational perspective. *Annual Review of Neuroscience*.

[19] Yazdi M., Khan F., Abbassi R., Rusli R. (2020). Improved DEMATEL methodology for effective safety management decision-making. *Safety Science*.

[20] Saydullaev S. R., Rahmatullaevich S. (2020). Decision-making system for the rational use of water resources. *Journal of Central Asian Social Research*.

[21] Yazdani M., Torkayesh A. E., Chatterjee P. (2020). An integrated decision-making model for supplier evaluation in public healthcare system: the case study of a Spanish hospital. *Journal of Enterprise Information Management*.

[22] Settembre-Blundo D., González-Sánchez R., Medina-Salgado S., García-Muiña F. E. (2021). Flexibility and resilience in corporate decision making: a new sustainability-based risk management system in uncertain times. *Global Journal of Flexible Systems Management*.

[23] Nemtinov V., Zazulya A., Kapustin V., Nemtinova Y. (2019). Analysis of decision-making options in complex technical system design. *Journal of Physics: Conference Series*.

[24] Hansen K. (2019). Decision-making based on energy costs: comparing levelized cost of energy and energy system costs. *Energy Strategy Reviews*.

[25] Fu M., Zhong Q., Dong J. (2022). Sports action recognition based on deep learning and clustering extraction algorithm. *Computational Intelligence and Neuroscience*.

[26] Ma X. (2022). Optimal control of whole network control system using improved genetic algorithm and information integrity scale. *Computational Intelligence and Neuroscience*.

